# A Computational Drug-Target Network for Yuanhu Zhitong Prescription

**DOI:** 10.1155/2013/658531

**Published:** 2013-05-09

**Authors:** Haiyu Xu, Ye Tao, Peng Lu, Peng Wang, Fangbo Zhang, Yuan Yuan, Songsong Wang, Xuefeng Xiao, Hongjun Yang, Luqi Huang

**Affiliations:** ^1^Institute of Chinese Materia Medica, China Academy of Chinese Medical Sciences, No. 16 Nanxiaojie, Dongzhimennei, Beijing 100700, China; ^2^Tianjin University of Traditional Chinese Medicine, Tianjin 300193, China; ^3^Institute of Automation, Chinese Academy of Sciences, Beijing 100190, China; ^4^Capital Medical University, Beijing 100069, China

## Abstract

Yuanhu Zhitong prescription (YZP) is a typical and relatively simple traditional Chinese medicine (TCM), widely used in the clinical treatment of headache, gastralgia, and dysmenorrhea. However, the underlying molecular mechanism of action of YZP is not clear. In this study, based on the previous chemical and metabolite analysis, a complex approach including the prediction of the structure of metabolite, high-throughput *in silico* screening, and network reconstruction and analysis was developed to obtain a computational drug-target network for YZP. This was followed by a functional and pathway analysis by ClueGO to determine some of the pharmacologic activities. Further, two new pharmacologic actions, antidepressant and antianxiety, of YZP were validated by animal experiments using zebrafish and mice models. The forced swimming test and the tail suspension test demonstrated that YZP at the doses of 4 mg/kg and 8 mg/kg had better antidepressive activity when compared with the control group. The anxiolytic activity experiment showed that YZP at the doses of 100 mg/L, 150 mg/L, and 200 mg/L had significant decrease in diving compared to controls. These results not only shed light on the better understanding of the molecular mechanisms of YZP for curing diseases, but also provide some evidence for exploring the classic TCM formulas for new clinical application.

## 1. Introduction

Traditional Chinese medicine (TCM) is one of the oldest systems of traditional medicines that make use of several herbs to cure a number of ailments for over 2,500 years [1, 2]. Recently, due to its good therapeutic effects and low toxicity, TCM has attracted considerable attention from all over the world [3]. However, the acceptance of TCM is restricted in the Western biomedical practice due to the lack of knowledge of mechanisms of action of the therapeutics as well as the characteristics of the active compounds. In the past, researches worked in the field of TCM had employed phytochemistry which also included separation, structure identification, and pharmacological research. However, those studies ignored the most essential features of multicomponents therapeutics and in turn the synergistic nature of TCM [4, 5]. The recent studies involving TCM have utilized system biology and network pharmacology to learn the molecular mechanism of TCM, such as TCM syndrome [6, 7], prescription compatibility [8], active substances and their pharmacological actions [9] et al. This approach provided deep understanding of TCM and improved the level of application, as well as promoted the modernization and globalization of TCM [10].

Yuanhu Zhitong prescription (YZP) is a typical and relatively simple TCM formula, consisting of *Radix angelicae dahuricae* and *Rhizoma corydalis* widely used in the clinical treatment of gastralgia, headache, and dysmenorrhea [11]. Alkaloids in *Rhizoma corydalis* and coumarins in *Radix angelicae dahuricae* are the active components in YZP [12, 13]. Recently, we developed a UPLC/Q-TOF-MS method to construct the chromatographic fingerprint and identify the 21 constituents of YZP [14]; we also developed an RRLC-QQQ technique to detect 17 constituents of YZP tablet [15]. Generally, only the absorbed constituents have more chances to play a role in the therapeutics. Thus, an RRLC-Q-TOF method was developed to identify 15 prototype compounds and some of their metabolites in plasma after oral administration of YZP extracts [16]. Pharmacologically, YZP has a wide variety of actions including antinociceptive [17], anti-inflammatory [18], spasmolysis [19], and vasorelaxation [20]; all of them may be the contributory factor for its therapeutic action. However, the molecular pharmacology of YZP is still unclear. The lack of the compound-target interaction network associated with YZP hindered the knowledge of molecular mechanism of YZP.

In this study, network pharmacology was employed as a tool to understand the active components in YZP and to know how YZP can be better administrated for its optimal therapeutic action. The objective of this study was to better understand the molecular mechanisms of YZP. Based on the known chemical and metabolic knowledge, an integrated model combining the metabolites' structure, virtual screening and validation of compound-target interaction *in silico*, network analysis, construction, and visualization, as well as bioactivity validation, had been performed to shed light on the mystery and effectiveness of YZP. 

## 2. Materials and Methods

The plan of work is depicted in Figure 1.

### 2.1. Database Construction

The constituents of YZP were derived from our earlier research on the analysis of the prototype constituents and the metabolites of YZP in the plasma [13]. Among them, 7 alkaloids were from *Rhizoma corydalis* and 8 coumarins were from *Radix angelicae dahuricae* (Figure 2). The molecular files of all prototype compounds were downloaded from ChemSpider (http://www.chemspider.com/) and saved to a mol format (molecular files). Six metabolites were identified by RRLC-Q-TOF and the Agilent Metabolite ID software (Agilent Technologies, Inc., 2009): 2 from tetrahydroberberine, 2 from tetrahydropalmatine, 1 from protopine, and 1 from oxypeucedanin (Table 1).

### 2.2. Prediction of Metabolites by Combined Computational Approaches

An ADMET predictor software program (ADMET Predictor, Simulations Plus, Inc., Lancaster, CA, 2012) was employed to predict atomic sites of metabolic reaction for CYP isoforms 1A2, 2C9, 2C19, 2D6, and 3A4. These isoforms account for ~90%–95% of CYP-mediated reactions. The mol files of molecular structure of oxypeucedanin, tetrahydroberberine, protopine, and tetrahydropalmatine were uploaded into the ADMET predictor software. The highest score of the metabolic “soft spot” was selected based on the metabolic type. These molecules were then exported as a mol file.

### 2.3. Molecular Similarity and Targets Identification

Drug data of 1447 FDA-approved drugs were collected from DrugBank database (http://www.drugbank.ca/, accessed on 2011.10.16). MedChem Studio (MedChem Studio, 3.0; Simulations Plus, Inc., Lancaster, CA, 2012.) could be powerful to quickly identify all molecules that are structurally similar to a reference molecule of interest. We used it to screen similar drugs of YZP by the comparison of 2D structural similarity between the ingredients of YZP (including 15 prototype constituents and 6 metabolites) *in vivo* and drug data. In order to improve the reliability of the results, only high similar drugs were selected according to the similar scores. All therapeutic targets of these similar drugs were also collected as predicted effector molecules of YZP.

### 2.4. Network Construction and Analysis

The 21 constituents of YZP were classified by 2D chemical structural similarity using MedChem Studio software program. The therapeutic similarity of the target (TST) was established based on anatomic therapeutic chemical (ATC) classification system corresponding to drug. The potential targets were identified based on the similarity of ATC codes corresponding to the drug by proposing a probabilistic model [21, 22]. The similarity between two ATC codes was derived according to their prior probabilities (frequency) and the probability of their commonality, which was defined as their longest matched prefix:

(1) S(atci,atcj)=2∗log⁡⁡(IC(prefix(atci,atcj)))log⁡⁡(IC(atci))+log⁡⁡(IC(atcj)),

where prefix (*i*, *j*) is the longest matched prefix of ATC code *i* and *j*. IC is the information content of ATC code. Note that drugs related to target may have more than one ATC code; we defined the maximum ATC code similarity as TST:

(2) $$\begin{array}{c} \text{Target}\;\;T_{1}\sim \text{ATC}\left(T_{1}\right)=\left\{{\text{atc}}_{11},{\text{atc}}_{12},\ldots ,{\text{atc}}_{1m}\right\},\\ \text{Target}\;\;T_{2}\sim \text{ATC}\left(T_{2}\right)=\left\{{\text{atc}}_{21},{\text{atc}}_{22},\ldots ,{\text{atc}}_{2n}\right\},\\ \text{TST}\left(T_{1},T_{2}\right)=\frac{\left|\text{ATC}\left(T_{1}\right)\cap \text{ATC}\left(T_{2}\right)\right|}{\left|\text{ATC}\left(T_{1}\right)\cup \text{ATC}\left(T_{2}\right)\right|}. \end{array}$$

ATC (*T*) represents all the ATC codes belonging to target corresponding to drug.

The potential targets were used to build the compound-target networks (CTN) with the 21 constituents of YZP. CTN was generated by Cytoscape 2.8.1, a standard tool for integrated analysis and visualization of biological networks, which was available for download from http://cytoscape.org/. In the graphical network format, nodes represent compounds or targets. Edges encode the compound-target and target-target interactions. From the relationship between chemical structural similarity and the therapeutic similarity, compound combinations and therapeutic targets, the qualitative properties of the networks were analyzed.

### 2.5. Functional and Pathway Analysis

ClueGO, Cytoscape plug-in, a professional software to facilitate the biological interpretation and to visualize the functionally grouped terms in the form of networks and charts [23], was used to perform functional and pathway analysis for the targets related to YZP. Simple text format of the targets in gene identifiers type was directly uploaded into the ClueGO software (Institute for Genomics and Bioinformatics Graz University of Technology, Graz, Austria). Enrichment/depletion tests were conducted for terms and groups as two-sided (enrichment/depletion) tests based on the hypergeometric distribution. The network type was selected as a “Medium” network. To create the annotations network, functional groups were visualized in the network using ClueGO which employed the organic layout algorithm.

## 3. Target Validation

The molecular docking simulation was further performed to validate the associations of candidate effector molecules with compositive compounds of YZP using eHiTS software program (Version 4.5, SimBioSys Inc., Canada). All the crystal structures of the targets were directly downloaded from RCSB protein data bank (http://www.pdb.org/, updated in 2012-6-11) and were carefully checked for their resolutions. The 3D structure of 15 prototype constituents was downloaded from ChemSpider in the mol files. The molecular structure of the metabolites was translated into 3D structure through CORINA, a fast and powerful 3D structure generator for small and medium sized molecules. A docking score calculated by the customizable scoring function of eHiTS, which combines novel terms (based on local surface point contact evaluation) with traditional empirical and statistical approaches, was used to measure the binding efficiency of each effector molecule to the corresponding compound [24]. While the docking score was lower than −5.0, these proteins were identified as candidate effector molecules which could bind their corresponding compounds with strong binding efficiency.

## 4. Bioactivity Validation

### 4.1. Animals and Housing

#### 4.1.1. Anxiolytic Activity

The anxiolytic activity of YZP was determined by using the AB line zebrafish (Danio rerio). Zebrafish were purchased from Harvard Medical School (Boston, MA, USA). The experiments were conducted at Biology Institute of Shandong Academy of Sciences. Zebrafish were kept at approximately 28°C on a 12 : 12 h light/dark cycle in an automated flow-through continuously filtered water system (Aquatic Habitats, Apopka, FL, USA). During the light phase, that is, between 8:00 a.m. and 8:00 p.m., the experiments were carried out to test the drug effect on the behavioral pattern of the Zebrafish. The fish were randomly sorted into treatment groups and vehicle-treated controls for the sake of avoiding any influence of breeding or holding conditions with drug treatment in the study. The tank water was prepared using mixing deionized H_2_O and sea salts (Instant Ocean, 1.2 g/20 liters of H_2_O). They were housed in 6-liter tanks and fed twice daily with flake fish food. The tanks were maintained under constant filtration and aeration.

#### 4.1.2. Antidepressant Activity

Male C57 black 6 mice were purchased from the Experimental Animal Center of Peking University Health Science Center, Beijing, China. Animals weighing at 18–22 g were housed in a breeding room at temperature of 22 ± 2°C, humidity of 60 ± 5%, and 12/12 h dark-light cycle. In order for the animals to adapt to the laboratory conditions, they were housed under those conditions for three days before starting the experiments. Tap water and food were provided ad libitum, but animals were fasted (with free access to water) before the experiments for 12 h. All possible steps were taken to avoid pain and discomfort to animals at every stage of the experiment. The animal experiments complied with the Guide for the Care and Use of Laboratory Animals (National Research Council of the USA, 1996) and related ethical regulations of China Academy of Chinese Medical Sciences.

### 4.2. Determination of Anxiolytic Activity

#### 4.2.1. Test Apparatus and Procedure [25, 26]

The Zebrafishes were placed in one of two plastic tanks with a capacity of 1.5 liter. The trapezoidal tanks (bottom: 22.9 cm, top: 27.9 cm, height: 15.2 cm, diagonal side: 15.9 cm) were filled with 1,350 mL of home tank water from the fish housing apparatus. It was 6.4 cm wide at the top and tapered to 5.1 cm at the bottom. The tanks were placed in such a way that the diagonal sides were facing each other, with a sheet of white paper blocking the view into the other tank. The tanks were back lit and had a translucent white sheet of plastic as the background so as to improve the performance of the imaging system. EthoVision (Wageningen, The Netherlands), a Samsung 8 mm camcorder, was used to record the image into the Noldus Image Analysis program. The tanks were positioned 88.5 cm from this camcorder. The Noldus software was applied to assess the swimming behavior (tank location choice). The index of anxiety was evaluated by the choice of position (bottom versus upper levels). Choice of dwelling on the bottom was near a position of safety similar to the position choice of closed versus open arms in the elevated plus maze and positions near the wall (thigmotaxis) versus the center of an open field with rodents. As with the elevated plus maze and open field in rodents there was a separate total activity measure as well.

#### 4.2.2. Drug Administration

In order to administer buspirone HCl (Sigma, St. Louis, MO, USA), Zebrafish were immersed in a beaker containing drug solution (25 mg/L) for 3 min. The extract of YZP was prepared according to the previous study [16] and administered at different concentrations (100, 150, and 200 mg/L) by immersing the Zebrafish for 3 min in a beaker containing YZP. A five-minute pause was obligatory between the end of dosing and the start of the experiment. The fish were exposed to the drug in a separate beaker and then were put into a holding tank without drug during this five-minute interval. For both buspirone and YZP, tank water was used as the vehicle. The control in this study was the exposure to tank water without the drug added. Home tank and the test chamber were completely devoid of any drug exposure. All the fish were drug naïve and each fish was used only once. There were at least 10 fish per condition.

### 4.3. Determination of Antidepressant Activity

The antidepressant activity was determined by the following behavioral tests: forced swimming test (FST), tail suspension test (TST), and locomotor activity measurement.

#### 4.3.1. Locomotor Activity Measurement

Locomotor activity was measured with locomotor activity system (YLS-1A, Yanyi Science and Technology Co. Ltd., Jinan, China). Animals were placed in the chamber of locomotor activity measurement device to adjust to the environment for 1 minute, followed by recording locomotor counter for 6 min.

#### 4.3.2. FST

The test was performed using the method reported by Porsolt et al. [27]. One hour after the last drug administration, each mouse was placed in an open cylindrical container (20 cm in height and 12 cm in diameter) filled with 12 cm of water (22 ± 1°C). A mouse was judged to be immobile when it remained floating in the water, making only the necessary movements to keep its head above water. The animals were constantly observed to ensure no contact between their paws and the base of the cylinder during FST [28].

#### 4.3.3. TST

This test was performed as described previously [29]. Briefly, 1 h after the last drug administration, animals were suspended by the tail from a ledge with adhesive tape (approximately 1 cm from the tip of the tail). The distance between the tip of tail and the floor was approximately 30 cm. Animals were partitioned to avoid interference during the test. Immobility was defined as the absence of movement and was scored over a 6 min trial by an observer blinded to the drug treatment.

#### 4.3.4. Drug Administration

Fluoxetine (30 mg/kg) and YZP at the doses of 4, 8, and 16 g/kg were administered to the mice. Fluoxetine (Fluox) was selected as positive control for depression and saline (0.9% NaCl) as control. Seventy-five mice (five groups of fifteen) were randomized into control and experimental groups. Animals in the control group received normal saline (0.9% NaCl). Animals in the three YZP treatment groups received the YZP at the doses of 4, 8, and 16 g/kg. Animals in the fluoxetine treatment group received fluoxetine at the dose of 30 mg/kg. All drugs and saline were administered i.g. in a volume of 20 mL/kg for seven days before the behavioral tests.

#### 4.3.5. Statistical Analysis

Data were expressed as mean ± standard error of mean (SEM) and analyzed using SPSS statistical software package. Statistical differences for experiments with more than three groups were determined by analysis of variance (ANOVA). For experiments with two groups, *t*-test was used. Differences were considered significant at *P* value less than 0.05.

## 5. Results and Discussion

### 5.1. Identification of Metabolites

Generally, most of TCM herbs are taken orally. It appears that compounds with assumed pharmacological value not only show a good target binding, but also have a chance to reach the target *in vivo*. Thus, detection and identification of the absorbed components and their metabolites are critical steps in the validation of the biological effect and the identification of the mechanism of action of TCM. In most cases, the metabolites play a crucial role in the curative effect. If followed by separation and structure identification, it is an extremely costly and time-consuming process especially for TCM herbs. In recent years, prediction tools based on *in vitro* and *in silico* input parameters have become more popular [30]. ADMET Predictor has emerged as a quick and useful tool to predict metabolic types and sites so as to confer the structure of the metabolites [31]. This comes from Simulations Plus, Inc, a leading provider of simulation and modeling software for pharmaceutical discovery. So far, based on the available evidence, the results would become more credible if combined with related experimental information [32]. Currently, an RRLC-Q-TOF MS/MS method coupled with Agilent Metabolite ID software was used to rapidly identify these metabolites and accurately speculate the reactive types of metabolism in our previous study. Afterward, ADME/T software has emerged as a quick and useful tool to predict metabolic types and sites so as to confer the structure of the metabolites.

In our previous study [16], 6 metabolites were detected *in vivo* and the types of reactions were concluded by RRLC-Q-TOF and the Agilent Metabolite ID software (Agilent Technologies, Inc., 2009) (Table 1). For example, demethylation reaction of tetrahydroberberine and tetrahydropalmatine happened and two metabolites were identified. Simultaneous demethylation and hydrogenation of protopine occurred and one metabolite was identified. Similarly, methylene to ketone of oxypeucedanin also took place and one metabolite was identified. Metabolic sites of four compounds were inferred by ADME/T software and the higher scores were selected. The structures of six metabolites (compound 16, 17, 18, 19, 20, and 21) were obtained (Figure 3).

### 5.2. Network Construction and Analysis

With the development of systems biology and the emergence of chemogenomic approaches, high-throughput virtual screening was found to be useful to better understand their possible molecular mechanisms. Recently, a number of computational methods have been developed for drug-target network predictions [33–38]. The similarity principles can be efficient complements for compound-target associations using similarity metrics such as ligand chemical similarity and drug side effects similarity [39]. The DrugBank database is a unique bioinformatics and cheminformatics resource that combines detailed drug data with comprehensive drug target information. Among them, 1447 FDA-approved small molecule drugs are selected and used to calculate the similarities with the constituents of YZP. Similar chemical structures are usually correlated with the therapeutic and pharmacological action [40, 41]. Furthermore, some methods have been developed to build the relationship between chemical structures and the therapeutics using the ATC classification system [42, 43]. In order to further understand the potential relationship between multicomponent and therapeutic effects, a network construction and analysis approach was used to visualize and analyze the interaction data. This approach helped capture the complexity in a simple, compact, and illustrative manner.

The C-T network consisted of 143 nodes and 1049 edges, including 21 candidate compounds (11 from *Rhizoma corydalis* and 10 from *Radix angelicae dahuricae*) and 122 candidate targets.  Figure 4 shows a global view of C-T network with color-coded and shape-coded nodes: compounds (green-lozenge) and candidate targets (purple-round). Complex networks are always very huge and have a distributed nature. Clustering is an important data-mining technique used to find data segmentation and pattern identification. Therefore, it is gradually becoming an instant requirement to propose fast network clustering algorithms in the sight of local view. Data showed that [44–46] similar compounds usually had similar therapeutic and pharmacological action. According to the chemical structure similarity, 21 compounds were classified into three categories: category I included protopine (Compound 15) and its metabolite (Compound 21), category II included the alkaloids (Compounds 7, 8, 11–14, and 17–20) and category III included all coumarins (Compounds 1–6, 9, 10, and 16). Targets were classified as many categories according to ATC classification system and main categories included dopamine receptors (DA) family, 5-hydroxytryptamine receptors (5-HT) family, alpha-adrenergic receptors (AA) family, gamma-aminobutyric acid receptors family, muscainic acetylcholine receptors (MA) family, phosphodiesterases family, inflammatory activator family for asthma, antibacterial effect family, and antitumor activity family. It was observed that different classes of compounds had some independent targets and the independent therapeutic effect. It was also observed that different classes of compounds had some common targets and therapeutics. But a lot of targets were clustered as a group alone.

Individually, most compounds might possess dozens of potential candidate targets, but a few compounds might have few candidate targets. Compounds 1, 13, 17, and 18 exhibited the highest number of candidate target interactions (73) followed by Compound 12 (with candidate targets of 42). Compound 10 had the least candidate targets (19) but its metabolite (Compound 16) had 34 candidate targets. Compound 7 had no candidate target.

YZP had been clinically used in TCM for the relief of pain, including headache, stomachache, and dysmenorrhea. In this study, C-T network might exhibit the synergy mode of “multicomponents, multitargets” and facilitate the understanding of the possible molecular basis of YZP therapeutic action. In our previous study [12], it was seen that most alkaloids of YZP can enter in the brain and can be bound with opioid receptors, DA receptors, 5-HT receptors, GABA receptors, and MA receptors. Tetrahydropalmatine and its metabolites are potential opioid antagonist drugs that had been clinically used for relief of pain [47]. In addition, DA receptors might coordinate motor functions and induce pain inhibition so as to relieve pain directly or indirectly [48]. Among AA receptors family, alpha 1 receptors are characteristics of vascular smooth muscle. Alpha 2 receptors are abundant in the brain and are associated with the pain perception [49]. Coumarins of *Rhizoma corydalis* can be primarily connected with the following targets groups: anti-inflammatory targets for asthma, drug targets for obstructive airway disease, antifungal receptors and sodium-dependent transporters, and DNA gyrase. Among them, anti-inflammatory targets for asthma can control chiefly airway responsiveness and reduce airflow resistance and asthma exacerbation [50]. Drug targets can be involved in bronchodilatory and anti-inflammatory effects for obstructive airway disease, which might be possibly related to the TCM theoretics of “regulating Qi.” It is still unclear that how the compound-target interaction of coumarins is responsible for its therapeutic action, which needs further research.

### 5.3. Molecular Functional and Pathway Analysis

Bioinformatics enrichment tools have played a very important and successful role contributing to the gene functional analysis for TCM biological studies. A number of high-throughput enrichment tools were independently developed as initial studies to address the challenge of functionally analyzing large gene lists [51]. As most of these tools mainly present their results as long lists or complex hierarchical trees, ClueGO, a Cytoscape plug-in, was developed to facilitate the biological interpretation and to visualize functionally grouped terms in the form of networks and charts [52]. The GO molecular function and Kyoto Encyclopedia of Genes and Genomes (KEGG) analysis for multitargets of YZP are shown in Figure 5(a). The main molecular functions were classified into seven categories: opioid receptor activity, GABA-A receptor activity, benzodiazepine receptor activity, DNA topoisomerase (ATP-hydrolyzing) activity, cholinesterase activity, dopamine receptor activity, and cation channel activity. The main pathways in KEGG were also classified into five categories as follows: linoleic acid metabolism, renin-angiotensin system, gap junction, ligand-receptor interaction, and calcium signaling pathway (Figure 5(b)).

In the practice of TCM, since long time, YZP has been used as an analgesic agent; some animal experiments indicated that YZP possesses the pharmacological action of analgesic [53, 54]. The present study indicated that YZP possesses multipharmacology molecular attributes through different target groups such as opioid receptors, dopamine receptors, and calcium channel. for pain relief. YZP activates opiate receptors to release met-enkephalin which stimulates the pleasure centers for analgesia [55]. Dopamine receptors, which are associated in many neurological processes, including motivation, pleasure, cognition, and memory, are also potential targets of YZP. The main constituents of YZP can pass through the blood brain barrier to exert a pharmacological action [16]. Calcium channel receptors and acetylcholine binding can play a crucial role in acute endothelium-dependent vasodilator responses to contract smooth muscle of the blood vessels and change arterial blood flow, which may explain their efficacy in migraine prevention [56].

In addition, a histamine receptor can inhibit gastric acid secretion, promote gastrointestinal motility, and relax gastrointestinal smooth muscle [57]. Cholinesterase receptors can relieve gastrointestinal smooth muscle spasm including the removal of vasospasm and improve microvascular circulation [58]. These could be the potential molecular mechanism by which YZP cures gastralgia.

YZP has the efficacy of “regulating Qi and invigorating blood circulation” in the practice of TCM [11]. In metabolic pathways of KEGG, most targets belonged to two families, linoleic acid metabolism and renin-angiotensin system. Linolenic acid metabolism is a very important metabolic pathway which has many biological effects, including potential immunomodulatory effects. This could change the platelet membrane fluidly, thus changing the number of platelet reactivity and platelet surface receptor stimulation. This in turn effectively prevents the formation of blood clots [59]. Renin-angiotensin system and hormonal regulation system of the human body have vital roles in the regulation of blood pressure, the balance of the electrolyte and fluid, and the development of the cardiovascular system [60].

Further, some new activities were found to be related with YZP, which might provide some evidence for new application of YZP. For example, many alkaloids were connected with GABA receptors group which suggested that YZP might possess anxiolytic action. Among them, dL-tetrahydropalmatine had been reported to have anxiolytic-like action [61]. It was also assumed that YZP might possess antidepressant action because of binding with benzodiazepine receptors in GO functional analysis (Figure 5(a)). Interestingly, YZP is supposed to have the molecular pharmacology of anticancer action by interaction with DNA topoisomerases which had been reported in the previous studies [62].

### 5.4. Target Validation

As a complementary medical system to Western medicine, TCM provides a unique theoretical and practical approach to the treatment of diseases over thousands of years. Natural products, containing inherently large-scale structural diversity more than synthetic compounds, have been the major resources of bioactive agents and will continually play as protagonists for discovering new drugs [63]. In order to better understand the profiles of compound-target interaction from the C-T network and provide an efficient approach to drug discovery, molecular docking is an established *in silico* tool used for searching the potentially highly bioactive compounds (Table 2). The results suggested that 17 pairs of compound-target interaction were found and their scores of docking were greater than 5. Similarly, some compounds had several candidate targets. Corydaline could be connected with four targets including CHRM2, CHRM3, ESR1, and DRD3. Protopine_M1 could be connected with 4 targets including ABCC8, BCHE, RNASE3, and KCNJ8. Tetrahydropalmatine could be connected with 3 targets including ADRA1A, OPRK1, and HRH1. But the other constituents had a single target. For example, *α*-allocryptopine had interacted with ESR2, tetrahydroberberine bound with ACE and oxypeucedanin bound with CRYZ.

### 5.5. Bioactivity Appraisal

The C-T interaction network and molecular functional analysis suggested that YZP had polypharmacologic actions which were integral to regulate the biological network of disease. Polypharmacologic actions included antinociceptive [17] and vasorelaxation [20]. As per our understanding, per computational biology, YZP has anxiolytic and antidepressant activity, which could be auxiliary therapy for headache and dysmenorrhea. The computational results indicated that the active constituents were not single but the mixture of multicompounds. Therefore, in the current study, YZP extract was used to validate the anxiolytic and antidepressant activities by animal experiments.

### 5.6. Assay of Anxiolytic Activity

Zebrafish are widely used in studying the molecular bases of neurobiology with applications in neuropharmacology and neurotoxicology [25, 26]. Bencan et al. [64] had developed a method to assess novel environment diving behavior of Zebrafish as a model of stress response and anxiolytic drug effects. Anxiety-like behavior in Zebrafish has been shown through patterns of swimming along the edge and towards the bottom of novel environments [65, 66]. The present study showed that buspirone at doses of 25 mg/L caused significant (*P* < 0.01) increases in diving compared to controls. Individually compared with control, YZP at doses of 100 mg/L, 150 mg/L, and 200 mg/L caused significant (*P* < 0.05, *P* < 0.01, and *P* < 0.01, resp.) decreases in diving. Even though low dose (100 mg/L) and middle dose (150 mg/L) showed dose-effect relation, there was no significant difference between middle dose and high dose (200 mg/L) (Figure 6). The results suggested that exposure to YZP treatment could reduce anxiety levels in Zebrafish.

### 5.7. Assay of Antidepressant Activity

Behavioral studies play an important role in the evaluation of antidepressant activity [66]. The FST and the TST are behavioral despair tests, useful for probing the pathological mechanism of depression and for the evaluation of antidepressant drugs [67] and had been widely used as preclinical screening tools for antidepressant drugs [68]. From the FST, it was seen that YZP at doses of 4 g/kg and 8 g/kg exhibited significantly (both *P* < 0.01) shorter duration of immobility and better antidepressive effect than that of fluoxetine (30 mg/kg) (Figure 7(a)). However, the highest doses (16 g/kg) did not show antidepressant activity. The TST results demonstrated that the immobility time was significantly lower in mice treated with YZP at the doses of 4 and 8 g/kg (*P* < 0.05 and *P* < 0.01, resp.) than mice in control group. However, the highest dose of YZP did not show any such effect (Figure 7(b)). In the FST and TST, false-positive results may exist with certain drugs, in particular psychomotor stimulants, which decrease immobility time by stimulating locomotor activity [69, 70]. Here, the locomotor activity of the mice was measured and the results suggested that YZP at different doses decreased locomotor counters in spontaneous motor activity (Figure 7(c)). These animal studies had revealed the antidepressant effect of YZP. It was also noted that the spontaneous motor activity was inhibited and the highest doses of YZP could not exhibit the antidepressant activity which may be due to the potential sedative activity related to GABA receptors.

## 6. Conclusions

TCM is regarded as an ancient, vital, and holistic system of health and healing, based on the notion of harmony and balance. Recently, network pharmacology emerged as a powerful tool to uncover molecular mechanisms and connections between the drug constituents and their targeting network. Currently, some researchers obtained the compounds from TCM database but they ignored the contents and pharmacokinetic profiles of the constituents, as well as their metabolites. In this study, 15 prototype constituents existed abundantly in YZP extracts and could be detected in the rat plasma and cerebrospinal fluid. At the same time, 6 metabolites were found *in vivo* and their structures were concluded successfully by high resolution of MS data and ADME/T software. An integrated compound-target interaction network of YZP was reconstructed through similar chemical structure searching based on the prototype compounds and their metabolites *in vivo*. The results of further network analysis based on ATC classification and GO molecular function indicated that similar compounds in YZP possess similar therapeutic action and share the similar pharmacological space. YZP exhibited the synergy mode of “multicomponents, multitargets” in the C-T network and possessed potential multipharmacologic activities. Importantly, many pharmacologic actions could be validated by the data and animal experiments. The findings helped to deeply understand the molecular mechanisms of YZP and also provided some evidence on new potential clinical application. Interestingly, YZP has the anxiolytic and antidepressant activities which would be worth developing and researching.

## Figures and Tables

**Figure 1:** Flowchart of the model building.

**Figure 2:** The structures of the 15 absorbed compounds and 6 metabolites of YZP: (1) imperatorin; (2) byakangelicol; (3) byakangelicin; (4) bergapten; (5) psoralen; (6) xanthotoxin; (7) coptisine; (8) *α*-allocryptopine; (9) isoimperatorin; (10) oxypeucedanin; (11) corydaline; (12) tetrahydropalmatine; (13) tetrahydroberberine; (14) berberine; (15) Protopine.

**Figure 3:** The possible metabolic sites and metabolites of six compounds: (16) tetrahydroberberine_M1; (17) tetrahydroberberine_M2; (18) tetrahydropalmatine_M1; (19) tetrahydropalmatine_M2; (20) protopine_M1; (21) oxypeucedanin_M1.

**Figure 4:** Compounds-targets (C-T) network. The C-T network is generated by linking the candidate compounds and all their candidate targets, with color-coded and shape-coded nodes: compounds (green-lozenge), candidate targets (purple-round).

**Figure 5:** (a) Functionally grouped network for the candidate targets of YZP. Functionally grouped network for the candidate targets of YZP with terms as nodes linked using ClueGO analysis, where only the label of the most significant term per group is shown. The node size represents the term enrichment significance. Functionally related groups partially overlap. (b) Pathway grouped network for the candidate targets of YZP. Pathway grouped network for the candidate targets of YZP with terms as nodes linked using ClueGO analysis, where only the label of the most significant term per group is shown. The node size represents the term enrichment significance. Functionally related groups partially overlap.

**Figure 6:** Anxiolytic-like effect of YZP. Anxiolytic-like effect of YZP (100 mg/kg, 150 mg/kg, and 200 mg/kg, resp.) on bottom dwelling (sec/min) in zebrafish (mean ± sem). Significant differences: *P < 0.05 and **P < 0.01, compared with the untreated control group.

**Figure 7:** Antidepressant-like effect of YZP. (a) Effects of YZP and fluoxetine (Fluox) on locomotor counters in locomotor activity. Significant differences: *P < 0.05 and **P < 0.01, compared with the untreated control group. (b) Antidepressant-like effect of YZP (4 g/kg, 8 g/kg and 16 g/kg, resp.) on the FST in mice. Animals were given i.g. YZP or fluoxetine before the tests. The duration of immobility in FST during the last 4 min of the test was recorded. No significant difference was found between Fluoxetine and YZP treated groups. Values were expressed as the mean ± SEM and analyzed using one-way ANOVA. Significant differences: *P < 0.05 and **P < 0.01, compared with the untreated control group. (c) Antidepressant-like effect of YZP (4 g/kg, 8 g/kg, and 16 g/kg, resp.) on the TST in mice. The duration of immobility in TST during the 6 min of the test was recorded. No significant difference was found between Fluoxetine and YZP treated groups. Values were expressed as the mean ± SEM and analyzed using one-way ANOVA. Significant differences: *P < 0.05 and **P < 0.01, compared with the untreated control group.

**Table 1:** Six metabolites of YZP detected *in vivo* from the previous experiment.

No.	RT (min)	[M + H]^+^	Formula	Metabolite name	Formula change	Parent compound	Source
M1	4.1880	342.1333	C_19_H_19_NO_5_	Demethylation, hydrogenation	−CH_2_+H_2_	Protopine	Plasma
M2	9.08278	342.1691	C_20_H_23_NO_4_	Demethylation	−CH_2_	Tetrahydropalmatine	Plasma
M3	10.6147	342.1695	C_20_H_23_NO_4_	Demethylation	−CH_2_	Tetrahydropalmatine	Plasma, CSF
M4	21.8366	301.0715	C_16_H_12_O_6_	Methylene to ketone	+O–H_2_	Oxypeucedanin	Plasma
M5	5.21887	326.1384	C_19_H_19_NO_4_	Demethylation	−CH_2_	Tetrahydroberberine	Plasma, CSF
M6	8.0093	326.1386	C_19_H_19_NO_4_	Demethylation	−CH_2_	Tetrahydroberberine	Plasma

CSF: cerebrospinal fluid.

**Table 2:** The eHiTS scores of potential targets.

NO	Gene name	PDB	Protein name	Compounds	eHiTS score
1	ESR1	1R5K	Estrogen receptor	corydaline	−6.99
2	DRD3	3PBL	D(3) dopamine receptor	corydaline	−6.53
3	CHRM2	3UON	Muscarinic acetylcholine receptor M2	corydaline	−6.33
4	CHRM3	4DAJ	Muscarinic acetylcholine receptor M3	corydaline	−6.28
5	CRYZ	1YB5	Quinone oxidoreductase	oxypeucedanin	−5.59
6	TOP2A	1ZXN	DNA topoisomerase 2-alpha	oxypeucedanin_M1	−5.79
7	VKORC1	3KP9	Vitamin K epoxide reductase complex subunit 1	byakangelicin	−6.04
8	ESR2	1QKM	Estrogen receptor beta	*α*-Allocryptopine	−6.13
9	ACE	1UZF	Angiotensin-converting enzyme	tetrahydroberberine	−5.69
10	ADRA1A	3SN6	Alpha-1A adrenergic receptor	tetrahydropalmatine	−5.97
11	OPRK1	4DJH	Kappa-type opioid receptor	tetrahydropalmatine	−5.57
12	HRH1	3RZE	Histamine H1 receptor	tetrahydropalmatine	−5.52
13	ADRA2A	3RFM	Alpha-2A adrenergic receptor	Tetrahydropalmatine_M2	−6.90
14	ABCC8	2BBO	ATP-binding cassette transporter subfamily C member 8	protopine_M1	−5.52
15	KCNJ8	3HFC	ATP-sensitive inward rectifier potassium channel 8	protopine_M1	−5.74
16	BCHE	2WIL	Cholinesterase	protopine_M1	−5.42
17	RNASE3	1DYT	Eosinophil cationic protein	protopine_M1	−5.21
